# An actin-dependent spindle position checkpoint ensures the asymmetric division in mouse oocytes

This article has been retracted.

**DOI:** 10.1038/ncomms8784

**Published:** 2015-07-15

**Authors:** Aïcha Metchat, Manuel Eguren, Julius M. Hossain, Antonio Z. Politi, Sébastien Huet, Jan Ellenberg

**Affiliations:** 1 European Molecular Biology Laboratory, Meyerhofstrasse 1, Heidelberg, Germany

## Abstract

Faithful chromosome segregation, during meiosis, is of critical importance to prevent aneuploidy in the resulting embryo. In mammalian oocytes, the segregation of homologous chromosomes takes place with the spindle located at the cell's periphery. The spindle is often assembled close to the centre of the cell, which necessitates the actin network for spindle transport to the cell cortex. In this study, we investigate how the segregation of chromosomes is coordinated with the positioning of the metaphase I spindle. We develop different assays to perturb the spindle's position and to delay its relocation to the cell periphery. We find that anaphase is delayed until the spindle is positioned in close proximity with the oocyte cortex. We further show that the metaphase arrest is dependent on a functional actin network, in addition to the spindle assembly checkpoint. Our work provides the first evidence for the existence of a functional spindle position checkpoint.

## Abstract (web summary)

In mammalian oocytes, the meiotic spindle is assembled close to the centre of the cell and relocates to the cell periphery prior to chromosome segregation. Here Metchat et al. show that anaphase is delayed until the spindle is positioned close to the cell cortex, providing evidence for a spindle position checkpoint.

Accurate chromosome segregation in mammalian oocytes requires chromosomes to achieve biorientation through the attachment of homologous kinetochores to the opposite poles of the meiotic microtubule spindle^1^,^2^,^3^,^4^. Errors in segregation of chromosomes during the first meiotic division, result in the generation of aneuploid embryos and cause pregnancy loss or severe birth defects such as Down's syndrome^5^,^6^,^7^. Similar to mitosis, the fidelity of chromosome segregation during oocyte meiosis is ensured by the spindle assembly checkpoint (SAC) which monitors kinetochore–microtubule attachment^2^,^3^,^8^,^9^,^10^,^11^,^12^,^13^,^14^,^15^,^16^,^17^. During meiosis I, all chromosomes usually achieve a stable biorientation 2–3 h before the onset of anaphase^1^,^4^. During this delay, a dynamic actin network spanning throughout the large cytoplasm moves the spindle from the centre toward the cortex of the oocyte^18^,^19^,^20^,^21^,^22^,^23^. The onset of anaphase coincides with the stable anchoring of the spindle, which allows the oocyte to divide asymmetrically (Fig. 1a). The spindle checkpoint protein Mad2 remains evident at kinetochores in late metaphase I, despite the fact that correct attachment of kinetochore fibres to the chromosome is achieved before spindle relocation^1^,^4^. These events suggest that chromosome biorientation may not be the sole mechanism that is monitored to prevent precocious chromosome segregation in oocytes. We hypothesized that SAC senses the spindle position in an actin-dependent manner to ensure the asymmetric division during meiosis I.

Here, we set out different assays to analyse whether the onset of chromosome segregation is linked to spindle position in mouse oocytes. Using these assays, we demonstrate the existence of a mechanism similar to the so-called ‘spindle position checkpoint' (SPC) in yeast^24^, which prevents chromosome segregation until the spindle is positioned in the cortical position.

## Results

### Quantitative analysis of spindle relocation

To quantitatively determine how the spindle is relocated from the centre to the cortex for chromosome segregation, we performed four-dimensional live-cell imaging of oocytes, in which microtubules were labelled with MAP4-GFP^1^,^25^, from the metaphase to anaphase stages using confocal microscope imaging (at 7-min intervals; Fig. 1b). To analyse our data, we developed an automated three-dimensional (3D) computational pipeline that detects the spindle on the basis of MAP4-green fluorescent protein (GFP) signal and uses the cytoplasmic background to precisely define the oocyte surface. This allowed us to measure the absolute distance between the spindle surface and the closest cortex, as well as the speed of relocation (Fig. 1c,d; Supplementary Fig. 1 and Supplementary Video 1). In addition, we computed the orientation of the spindle in 3D with respect to its initial orientation and the oocyte surface. Consistent with previous studies, the spindle formed in the centre of the oocyte (Fig. 1e). The metaphase I spindle is occasionally formed closer to the cortex because of the slight asymmetric position of the germinal vesicle^26^. At the onset of chromosome segregation, the shortest distance between the spindle surface and the cortex was 3.06±1.27 μm (mean value±s.d.). This distance corresponded to the enriched actin network between the cortex and the spindle surface^27^ (Fig. 1e). The meiotic spindle relocated to the cortex through three different phases (phases I, II and III). During phase I, the spindle started migrating at a low but progressively increasing speed from the centre to a location 9 μm away from its final position. During phase II, at 9 and 5 μm from its final position, the spindle migrated at its maximum speed. Upon arrival at the cortex in phase III, the displacement speed of the spindle decreased significantly (Fig. 1f,g). Next, to quantitatively determine whether the spindle kept the same orientation during its relocation, we defined the spindle axis using the principal component of segmented spindle voxels and measured the rotational movement of the spindle axis from the onset of migration to its arrival at the cortex (<5 μm; Fig. 1h,i and Supplementary Fig. 1). The average rotational movement of spindle orientation was 16.44°, indicating that spindle orientation does not change considerably during its relocation to the cortex (Fig. 1i). This finding is supported by previous observations that the spindle is pulled to the cortex through an interaction between the actin network and the closest spindle pole^18^,^19^,^20^,^28^. To determine whether the time of anaphase onset depends on the initial position of the spindle, we analysed the correlation between the initial distance between the spindle surface and the cortex and the time of chromosome segregation. We found that the initial spindle distance from the cortex correlates with the time delay of anaphase (*r*=0.78; Fig. 1j).

During meiosis I, anaphase entry is activated by anaphase-promoting complex (APC/C) that targets the key meiotic substrates for degradation, including Securin^11^,^12^,^29^,^30^,^31^,^32^. To understand the link between APC/C-mediated Securin degradation and spindle position, we quantitatively measured the Securin degradation during spindle relocation by live-cell imaging of oocytes expressing Securin-EGFP and H2B-mCherry. Interestingly, Securin degradation started only when the chromosome was located close to the cortex (distance between the centre of mass of chromosome and the cortex inferior to 20 μm, Fig. 1k,l). These data support the hypothesis that homologous chromosome segregation is coordinated with the asymmetric spindle position.

### Functional SPC during meiosis I

It has long been proposed that cortical positioning is not required for chromosome segregation during meiosis I. Depolymerization of the actin network by cytochalasin D (CD), which inhibits spindle relocation, does not affect the timing of chromosome segregation^21^,^33^. We obtained similar results using low-dose CD or latrunculin from metaphase I onward (Supplementary Figs 2a,b and 3a). Interestingly, actin-filament stabilization by jasplakinolide also had no effect on the timing of chromosome segregation compared with CD/latrunculin treatment, consistent with the findings of other reports on actin network perturbations^21^,^33^,^34^,^35^ (Supplementary Fig. 3b). To examine how APC/C is activated in CD-treated oocytes; we recorded the destruction of Securin at late metaphase stage. We found that the dynamics of Securin degradation in CD-treated oocytes was comparable with the control oocytes (Supplementary Fig. 2c).

We hypothesized that the dynamic actin network is the key sensor of spindle position. To test this hypothesis, we first depolymerized the actin filaments in metaphase I using low-dose CD, then removed the drug to nucleate the actin network *de novo* immediately before the expected time of chromosome segregation, that is, ∼7 h after germinal vesicle breaks down (GVBD; termed ‘SPC assay I'; Supplementary Fig. 4a). We observed that in CD-washout conditions, chromosome segregation was always preceded by the relocation of the spindle to the cortex (20/20 oocytes), with a significant delay in anaphase onset (1 h 34 min) compared with control oocytes (Fig. 2a–c; Supplementary Fig. 4b). In oocytes treated with CD long term, that is, in the complete absence of the actin network, chromosome segregation occurred at the same time as in control oocytes.

It has been shown in zebrafish oocytes that Cyclin B level is dependent on the actin network^36^. To investigate the actin-depolymerization effect on the endogenous level of Cyclin B, we immunostained Cyclin B in CD-treated oocytes immediately after the drug washout in SPC assay I. Cytoplasmic Cyclin B level in CD-treated oocytes was similar to control oocytes, showing that the delay of anaphase onset was not a consequence of Cyclin B level perturbation at late metaphase stage (Supplementary Fig. 4c,d). This result shows that repolymerization of the actin network delays chromosome segregation until the spindle reaches the cortex (Fig. 2b and Supplementary Fig. 4b).

To examine whether reassembly of the actin network inhibits chromosome segregation, we developed an assay for F-actin regrowth before and after spindle migration in synchronized oocytes (designed ‘SPC assay II'). Oocytes were transferred before or after spindle relocation to medium enriched with CD (Supplementary Figs 2a–5a). In addition, we used the proteasome inhibitor MG132 to prevent chromosome segregation during CD treatment. The timing and location of chromosome segregation was monitored after drug washout using live-cell imaging. Chromosome segregation occurred earlier when the spindle was already positioned at the cell periphery. For oocytes treated with CD before spindle relocation, the onset of anaphase only occurred when the spindle reached the cortex, causing a significant time delay (Supplementary Fig. 5b,c). These results indicate that the repolymerization of actin filaments does not directly affect chromosome segregation. It should be noted that these assays (SPC assays I and II) were conducted without micro-manipulating the oocytes. Therefore, the time delay observed was not due to artifactual spindle disruption. Taken together, these data showed that an F-actin-dependent mechanism delays the onset of anaphase until the spindle is correctly positioned near the cortex.

### Spindle motion and orientation in SPC assay

To further study the relationship between spindle displacement and chromosome segregation, we developed an assay on the basis of oocyte centrifugation using Maro chamber in order to shift the position of the spindle (termed ‘SPC assay III'; Supplementary Fig. 6a; Fig. 3a,b and Supplementary Video 2). The computational pipeline, described in Supplementary Fig. 1, was used to analyse spindle displacement. After centrifugation, the spindle was displaced from the centre to a random position in the cytoplasm. During SPC assay III, the spindle first moved to the cortex, an event followed by chromosome segregation (42/43 oocytes, Fig. 3c). Movement of the spindle toward the cortex occurred in three phases (phases I, II and/or III) depending on their initial distance from the cortex. When the distance from the cortex was large (11.05±1.17 μm), movement occurred successively through phases I, II and III, or I and II. When the distance between the spindle and its final position was 6.54±2.05 μm, the movement of the spindle started directly from phase II followed by phase III. In oocytes in which the spindle was located close to the cortex (3.85±1.02 μm), relocation only occurred via phase III (Fig. 3d). The maximum speed of migration was higher after MG132/CD washout, which explained the shorter duration of spindle relocation (Figs 1f and 3d). Analysis of spindle orientation showed that the spindle maintained its initial orientation during relocation (Fig. 3e). As before, we verified whether the endogenous level of Cyclin B was affected by the centrifugation. The level of Cyclin B in centrifuged oocytes was similar to that in non-centrifuged oocytes (Supplementary Fig. 6b). These data collectively show that the initial position and orientation of the spindle defines its subsequent speed and direction of motion.

### Actin network in SPC assay

To better understand the effect of actin filaments on the timing of chromosome segregation and the correct reconstruction of the meshwork in CD-washout oocytes, we imaged F-actin in live oocytes using the actin-filament marker EGFP-Utrophin after CD-washout (Supplementary Video 3)^18^,^19^,^20^,^37^. Reassembly of actin filaments was first detected on the spindle surface 10 min after drug washout and proceeded to the spindle's interior after a further 10 min (Supplementary Fig. 7a,b). Maximal length of actin filaments was achieved 20 min after drug washout (Supplementary Fig. 7c). The density of F-actin was higher in CD-washout oocytes than in control oocytes. Whether actin was functional after drug washout was investigated by tracking vesicles labelled with Rab11a-mCherry^34^,^38^. The maximum speed of vesicle displacement was achieved 20 min after CD-washout, indicating that the actin network is almost instantly reconstituted and functional during SPC assay (Supplementary Video 4; Supplementary Fig. 8a,b).

Our group and others have shown that the spindle motion requires direct interaction between F-actin filaments and the spindle poles. Using high-resolution imaging, we could observe that long actin filaments were present within the spindle. On the basis of these observations, we addressed the question whether these actin filaments, named spindle actin filaments, connect directly with chromosomes during the spindle motion. To this end, we imaged F-actin and chromosomes during the spindle migration in fixed oocytes using very high-resolution imaging. We observed several actin filaments surrounding chromosomes from the centromeric regions to the chromosome arms (Supplementary Fig. 9).

### SPC requires the SAC activity

The SAC regulates chromosome segregation by monitoring the kinetics of kinetochore biorientation and the correct attachment of kinetochore fibres^3^,^8^,^39^,^40^. Our data showed that the binding of SAC proteins persists even after chromosome biorientation during spindle relocation, consistent with the findings of previous studies^1^,^2^,^4^,^40^. To investigate whether metaphase arrest in the SPC assay was owing to SAC activity, we used Cdc20 with a point mutation, Cdc20^R132A^, which cannot bind to Mad2 (refs 31, 41, 42) (Fig. 4a and Supplementary Fig. 10). In Cdc20^R132A^-injected oocytes, chromosome segregation occurred before or during spindle relocation, resulting in the formation of a large polar-body or symmetric division (Fig. 4b–e). Next, to inhibit the SAC activity from metaphase I onward, we used reversine, a small molecule inhibitor of SAC, during centrifugation in the last step of the SPC assay. Reversine inhibits the kinase Mps1, a known positive regulator of the SAC upstream of Mad2 during meiosis and mitosis (Supplementary Fig. 10)^2^,^14^,^15^,^43^,^44^,^45^. In reversine-treated oocytes, chromosomes segregated before or at the onset of spindle relocation, resulting in the formation of a large polar-body or symmetric division, similar to Cdc20^R132A^-injected oocytes (Fig. 4f–h; Supplementary Video 5).

To confirm these results, we used dominant negative Mad2^ΔC^ to directly prevent Mad2 activity on kinetochores (Supplementary Fig. 11). After its recruitment to kinetochores, Mad2^ΔC^ binds to the endogenous Mad1–Mad2 core complex, inhibiting Mad2-Cdc20 binding^33^. As observed in our previous examinations of SAC perturbations, chromosome segregation occurred before or at the onset of spindle relocation, resulting in the formation of a large polar-body or symmetric division, in Mad2^ΔC^-injected oocytes compared with control oocytes (Supplementary Fig. 12a–c). These results showed that SPC requires Mad2 activity on kinetochores.

Previously, we showed that after chromosome biorientation, Mad2 bound 20–40% of kinetochores, which corresponded to the relocation of the spindle. To verify whether the delay in anaphase onset is likely due to the enrichment of Mad2 on kinetochores, we imaged non-centrifuged oocytes expressing Mad2-EGFP and H2B-mCherry after CD/MG132 washout. As expected, Mad2-EGFP marked 10–30% of kinetochores, at the onset of the spindle motion. We found that Mad2 is only delocalized from kinetochores after cortical positioning, suggesting that the maintenance of SAC activity may be due to the spindle motion (Supplementary Fig. 12d–f). Actin-filament repolymerization was verified by imaging Rab11a-mCherry positive vesicle dynamic in reversine-treated and Mad2-inhibited oocytes. We found that the mean speed of vesicle movement was similar in all culture conditions, indicating that the actin network was correctly repolymerized (Supplementary Fig. 13a–c). All these results reveal that SPC requires the SAC pathway via Mps1, Mad2 and Cdc20.

## Discussion

Our data showed that the metaphase I spindle moves to the cortex in three phases. In phase I, after bipolarization of the spindle, it moves slowly toward the closest cortex. Next, in phase II, the speed of displacement increases exponentially until it reaches a maximum, with the spindle in a specific spatial position. This increase in speed is correlated with the enrichment of actin filaments on the spindle pole during relocation. Finally, in phase III, the spindle finishes its journey by significantly decreasing its speed until it becomes stationary. Subsequently, chromosome segregation occurs. In the SPC assay, we shifted the spindle from its initial position to a random position in the cytoplasm by gentle centrifugation. We observed that, depending on its initial distance from the cortex, the spindle started its motion in phases I, II or III. These results suggest that the increase in velocity during relocation depends on the initial distance of the spindle from the cortex. The number of F-actin filaments attached to the spindle pole and the number of actin branches connecting the spindle to the cortex define the speed of relocation. This is supported by a recent elegant study combining *in vitro* manipulation and mathematical modelling, showing a link between the spindle position, the F-actin density and the pulling force^28^.

We proposed that the spindle position via the dynamic actin network determines the timing of chromosome segregation. In our previous study, we showed that chromosome biorientation occurs in four phases. During the first three phases, chromosomes and kinetochores move to the surface of the microtubule ball, undergo congression to yield the prometaphase belt, and become bioriented with the barrel-shaped bipolar spindle formation^1^,^2^. In phase IV, chromosomes are stably bioriented and positioned on the metaphase plate but continue to show low-amplitude oscillations. At this stage, Mad2 binds the kinetochore and the spindle starts migration toward the cortex. We speculate that force-driven spindle movement maintains SAC activity on kinetochores, creating a ‘wait-anaphase' signal. At the cortical position, the spindle stops moving; subsequently, all forces applied to the spindle pole are equal, and chromosome oscillation is interrupted. Next, Mad2 completely dissociates from the kinetochores, and APC/C mediates Securin degradation followed by the onset of anaphase. A study, using a different mouse strain, reported that chromosome biorientation completes immediately before the onset of anaphase. In the representative illustration of the experiment shown in this article, chromosomes are already positioned near the cortex during spindle formation and chromosome biorientation. Future studies should investigate, in mouse strains in which the spindle is often formed near the cortex, whether the delay in chromosome segregation after biorientation is systematically suppressed^2^.

In the last two decades, numerous studies have identified proteins involved in the regulation of actin network dynamics and spindle relocation. One representative protein is Mos, the mutation of which inhibits mitogen-activated protein kinase activity and spindle relocation, but does not interfere with polar-body extrusion^22^,^27^,^33^. A recent study reported that, in addition to these events, cortex softening is disturbed in *mos*^−/−^ oocytes^18^,^21^. In contrast, Formin-2, an actin nucleator and contributor to asymmetric spindle positioning, plays an essential role in cytoplasmic actin nucleation but does not regulate cortical actin. Similar to other actin perturbations, the timing of polar-body extrusion is unaffected in *Formin-2* and *Mos* mutant oocytes. These findings support our results, and suggest that both cortical and cytoplasmic actin are important for spindle position sensing.

Here, we showed that the regulation of chromosome segregation in vertebrate oocytes is more complex than a ‘biological clock' and the asymmetric spindle positioning combined. For the first time, we reveal the existence of a SPC, based on the activity of the SAC, alongside a dynamic actin network. In addition to the mechanical model involving actin and the SAC pathway, other factors may be involved in the regulation of the SPC and remain to be discovered.

## Methods

### Culture and micromanipulation of oocytes

Ovaries were collected from 8-week-old FVB or CAGH2BEGFP mice that were maintained according to the guidelines of EMBL laboratory animal resources, 44–48 h after priming with 5 IU pregnant mare serum gonadotropin. Oocytes were isolated by puncturing the ovaries with needles in M2 medium supplemented with 100 nM of IBMX (3-isobutyl-1-methylxanthine). To induce resumption of meiosis, oocytes were incubated in IBMX-free medium. In some experiments, the medium was supplemented with low concentration of CD (0.5 μg ml^−1^) and MG132 (4 μM) to prevent spindle relocation and chromosome segregation. To inhibit the activity of Mps1, oocytes were treated with reversine (an inhibitor of Msp1, 1.5 μM). In control, medium was supplemented corresponding amounts of DMSO (dimethyl sulfoxide). Microinjection of *in vitro*-transcribed RNAs to the oocytes was performed with 5 pl EB3-mCherry, 5 pl mCherry-H2B, 5 pl EGFP-MAP4, 1 pl Mad2-EGFP, Rab11a-mCherry, Cdc20^R132A^ and Mad2^ΔC^ of 1–2 μg μl^−1^ mRNAs.

### Immunofluorescence

Oocytes were fixed for 30–60 min at 37 °C in 100 mM HEPES (pH7; titrated with KOH), 50 mM EGTA (pH7; titrated with KOH), 10 mM MgSO_4_, 2% formaldehyde (methanol free) and 0.2% Triton X-100. Oocytes were left in PBS (phosphate-buffered saline) with 0.1% Triton X-100 overnight at 4 °C. F-actin staining was carried out in PBS with 0.1% Triton X-100 and 3% bovine serum albumin with Alexa-Fluor-488–Phalloidin (Molecular Probes, A12379; 1:100). DNA was stained with 5 mg ml^−1^ Hoechst 33342 or DAPI (Molecular Probes). As primary antibodies, we used mouse Cyclin B (Abcam, ab2949; 1:100). As secondary antibodies, we used Alexa-555-labelled goat anti-mouse (Life technologies, A21422; 1:500).

### Confocal microscopy

Images were acquired with a customized Zeiss LSM780 or Meta 510 confocal microscope, using a 40x C-Apochromat 1.2 NA water immersion objective lens. We recorded spindle and chromosomes dynamics by time-lapse (4D) imaging. For 10 cells in parallel, we imaged 25 z-confocal sections (every 3 μm) every 7 min for 5–10 h, which covers spindle migration to anaphase onset of meiosis I.

For spindle tracking with MAP4-EGFP and EB3-mCherry, we imaged 25 z-confocal sections (every 3 μm) of 512 × 512 pixel xy images, in total covering at least 70 μm × 70 μm × 75 μm volume, at time interval of 7 min for 10 h from early metaphase stage or after drug washout.

For Mad2-EGFP, we imaged 17 z-confocal sections (every 2.0 μm) of 512 × 512 pixel xy images, in total covering a 37.5 μm × 37.5 μm × 34.0 μm volume, at time interval of 10 min from 1 to 6 h after drugs washout, covering the spindle migration.

### SPC assay I

Oocytes expressing H2B-EGFP were collected at GV stage. After scoring GVBD, oocytes were transferred in M2 medium supplemented with 0.5 μg.ml^−1^ of CD. At the time of anaphase onset (7 h after GVBD), oocytes were transferred CD-free medium into the microscope to score the location and the time of chromosome segregation in non-treated (DMSO), CD-treated and CD-treated washout oocytes (Supplementary Fig. 4).

### SPC assay II

To induce maturation, fully-grown oocytes were incubated in IBMX-free medium. After scoring GVBD, synchronized oocytes were transferred in medium supplemented with low dose of CD (0.5 μg.ml^−1^) at metaphase I stage before or after spindle relocation. In addition, all oocytes were treated with low dose of MG132 (4 μM, an inhibitor of the proteasome) to prevent chromosome segregation by inhibiting Securin/Cyclin B degradation. MG132 was added at the late metaphase I to avoid any damage on the spindle steady-state. After drugs washout, oocytes were immediately transferred into the microscope to score the position and the time of chromosome segregation. The time of anaphase has been calculated between the drug washout and the onset of chromosome segregation (Supplementary Fig. 5).

### SPC assay III

Oocytes expressing H2B-EGFP were collected at GV stage, microinjected with 5 pl of EB3-mCherry and transferred immediately in IBMX-free medium. Two hours after GVBD, oocytes were treated with CD (0.5 μg ml^−1^). Seven hours after GVBD, oocytes were either treated with MG132 (4 μM) or MG132 combined with reversine (1.5 μM). Oocytes were transferred in Maro chamber positioned in 50 ml conical tube; and centrifuged for 1 h at 1,000 r.p.m. at 37 °C. After the centrifugation, oocytes were then released into MG132- and cytochalasin-D-free medium and transferred into the microscope for 4D live imaging (Supplementary Fig. 6).

### Spindle position and orientation tracking

To measure the kinetics of spindle relocation, we injected oocytes with mRNA encoding EB3-mCherry to label microtubules. We then imaged the entire oocyte volume during spindle relocation using an autofocussing macro (25z sections; spacing: 3 μm, time interval: from 7 min, maximum total duration: 10 h; parameters vary slightly in some experiments). Drifts during image acquisition were corrected with the ‘3D drift correction' function of Fiji. The cytoplasmic background has been enhanced using filtering (Gaussian blur) and Image Calculator in Fiji (http://rsb.info.nih.gov/ij/).

### Rab11a-mCherry vesicle tracking

Three-dimensional data sets of vesicles were acquired using Zeiss's Multi Time Series macro (13 sections; spacing: 1.5 μm; time interval: 6.3 s; total duration: ∼1 min). For peak enhancement of vesicle signals and background subtraction, vesicle images processed by a 10-pixel Gaussian blur were subtracted from the same images processed by a 2-pixel Gaussian blur. Drifts during image acquisition were corrected with the ‘Correct 3D drift' function of Fiji using the transmitted light. Vesicles were tracked using Imaris 3D spot tracking and the mean speed was calculated over 1 min. Average, s.d., and statistical significance based on Student's *t*-test were calculated in SigmaPlot software.

### Measurement of the cytoplasmic actin network density and actin-filament length

To measure the average filament length between two nodes, we recorded time-lapse imaging of oocytes expressing EGFP-UtrCH (time interval: 1 min) few minutes after the drug washout. The filament length between two nodes or between a node and the end of the filament in the cytoplasm was measured using Fiji. To measure the actin-filament density, the cytoplasmic background has been subtracted using filtering by Fiji software after the CD washout.

### Statistics

Average (mean), s.d. and statistical significance based on Student's *t*-test (always two tailed) were calculated in Excel and SigmaPlot. The sample size was chosen on the basis of Student's *t*-test. The end of all boxes plot defines the 25th and 75th percentiles, with a line at the median and error bars defining the 10th and 90th percentiles. The 2D and the 3D plots were generated by the plotting software Python (xy) (http://code.google.com/p/pythonxy/) or SigmaPlot software.

## Additional information

**How to cite this article:** Metchat, A. *et al*. An actin-dependent spindle position checkpoint ensures the asymmetric division in mouse oocytes. *Nat. Commun.* 6:7784 doi: 10.1038/ncomms8784 (2015).

## Supplementary Material

Supplementary Information Supplementary Figures 1-13

Supplementary Movie 1 Quantitative image analysis. Image segmentation of maturing oocyte expressing MAP4-GFP during spindle relocation.

Supplementary Movie 2 Spindle position checkpoint assay III. 4D live imaging of oocyte expressing H2B-GFP and EB3-mcherry, 20 min after the drugs washout.

Supplementary Movie 3 Actin repolymerization in spindle position checkpoint assay. Time-lapse imaging of oocyte expressing EGFP-UtrCH after CD-washout.

Supplementary Movie 4 Vesicle dynamics in spindle position checkpoint assay. Tracking of Rab11a-mcherry positive vesicles after CD-washout.

Supplementary Movie 5 Mps1 inhibited oocyte in spindle position checkpoint assay. 4D live imaging of oocyte expressing H2B-GFP and EB3-mcherry treated by low dose of Reversine, 20 min after the drugs washout.

## Figures and Tables

**Figure 1:** Complete 3D spindle movement tracking during meiosis I. (**a**) Schematic representation of meiosis I in mouse oocytes. (**b**) Time-lapse imaging of the spindle migration in live oocyte expressing MAP4-GFP (spindle in red). Scale bar, 10 μm. (**c**,**d**) Image reconstructed in 3D with Amira software representing segmentation of the spindle (in green) and the cortex (in white). (**e**) Histogram representing initial and final distance of spindle from the cortex in oocytes. (**f**) Average of spindle displacements (time alignment by cross correlation). The distance of the spindle surface from the closest cortex is plotted over time. The colour code showed the speed of displacement (in grey, the s.d.). The speed scale of spindle displacement is indicated by the colour bar. (**g**) The mean of the spindle speed was plotted over distance from the cortex (>3 independent experiments, *n*=21). (**h**) Three-dimensional reconstruction with Amira image of oocyte showing the orientation-deviation measurement during spindle relocation. (**i**) Histogram of angle deviations of spindle orientation during relocation (*n*=14). (**j**) The time of chromosome segregation is plotted over the initial distance of the spindle from the cortex (Pearson coefficient of correlation (*r*)=0.78 and *P*<0.001). (**k**) Time-lapse imaging of live oocyte expressing Securin-GFP and H2B-mCherry during spindle migration (securin in green, chromosomes in red), scale bar, 10 μm. (**l**) Average of normalized Securin-GFP fluorescence from metaphase stage to anaphase. The line corresponds to the time of the cortical positioning (in grey, the s.d., two independent experiments, *n*=6). Data are mean, with error bars displaying s.d. *P*-values were calculated with Student's test (nonparametric test, two tailed).

**Figure 2:** SPC assay I. (**a**) Two hours after GVBD, maturing oocytes were transferred into a medium containing 0.5 μg ml^−1^ of CD. At the expected time of chromosome segregation (7 h after GVBD), oocytes expressing H2B-EGFP were washed out from CD and transferred to the microscope for 4D live-cell imaging to record the time of anaphase. (**b**) Time-lapse imaging of chromosome segregation in control, CD-treated and CD-treated washout oocytes. Scale bar, 10 μm. (**c**) Time of chromosome segregation (GVBD-anaphase) in CD-treated (three independent experiments, *n*=24, *P*<0.001), CD-treated washout (three independent experiments, *n*=20, *P*=0.8) and control oocytes (three independent experiments, *n*=20). Data are mean, with error bars displaying s.d. *P*-values were calculated with Student's test (nonparametric test, two tailed).

**Figure 3:** SPC assay III. (**a**) Schematic representation of the SPC assay III. Two hours after GVBD, the oocytes were transferred into a medium containing 0.5 μg ml^−1^ of CD. At the expected time of chromosome segregation (7 h after GVBD), oocytes were transferred into medium containing 4 μM MG132 and 0.5 μg ml^−1^ of CD, centrifuged for 1 h at 1,000 r.p.m. at 37 °C. After the spindle shift, oocytes were immediately removed from CD and MG132 and transferred to the microscope for 4D live-cell imaging (details are shown in Supplementary Fig. 6a). (**b**) Time-lapse imaging of oocytes expressing EB3-mCherry and H2B-EGFP in the SPC assay III. On the top panel, the spindle was initially localized in the centre and on the bottom panel the spindle was localized close to the cortex. Scale bar, 10 μm. (**c**) Histogram representing initial (at the drugs washout) and final distance (at anaphase onset) of spindles from the cortex in oocytes after CD/MG132 washout in SPC Assay III (>3 independent experiments, *n*=43). (**d**) Quantitative analysis of the spindle displacement in the SPC assay III. (**e**) Histogram representing the angle deviation of the spindle orientation during the relocation.

**Figure 4:** SAC depletion inhibits SPC. (**a**) Protocol of SAC inhibition by Cdc20^R132A^ microinjection combined with the SPC assay. (**b**) Time-lapse imaging of Cdc20^R132A^-injected and control oocytes expressing EB3-mCherry (microtubule) and H2B-EGFP (chromosome) after CD/MG132 washout. Three-dimensional projection of the oocyte (white) and spindle (green) with Amira software from oocytes at the onset of anaphase. (**c**) Quantitative analysis of the spindle displacement, (**d**) initial (at the drug washout) and final distances (at anaphase onset) from the cortex (*P*<0.0001 in control oocytes, *P*=0.0462 in Cdc20^R132A^-injected oocytes) and (**e**) time of anaphase after the drugs washout in control (*n*=15, in black) and Cdc20^R132A^-injected oocytes (three independent experiments, *n*=18, in red, *P*<0.0001). (**f**) Dynamic of spindle relocation, (**g**) initial and final distance from the cortex (*P*<0.0001 in control oocytes and *P*=0.31 in Reversine-treated oocytes) and (**h**) time of anaphase after the drugs washout (two independent experiments, *n*=8, in black) in control and in reversine-treated oocytes (two independent experiments, *n*=8, in red; *P*<0.0001). Scale bar, 10 μm. Data are mean, with error bars displaying s.d. *P*-values were calculated with Student's test (nonparametric test, two tailed).
